RETRACTED

# Inflammatory-Related P62 Triggers Malignant Transformation of Mesenchymal Stem Cells through the Cascade of CUDR-CTCF-IGFII-RAS Signaling

**DOI:** 10.1016/j.omtn.2018.03.002

**Published:** 2018-03-09

**Authors:** Xiaoru Xin, Chen Wang, Zhuojia Lin, Jie Xu, Yanan Lu, Qiuyu Meng, Xiaonan Li, Yuxin Yang, Qidi Zheng, Xin Gui, Tianming Li, Hu Pu, Wujun Xiong, Jiao Li, Song Jia, Dongdong Lu

**Affiliations:** 1 Research Center for Translational Medicine at Shanghai East Hospital, School of Life Science and Technology, Tongji University, Shanghai 200092, China; 2 Department of Hepatology, Shanghai East Hospital, Tongji University School of Medicine, Shanghai 200120, China; 3 School of Medicine, Tongji University, Shanghai 200092, China

**Keywords:** P62, TNF-α, inflammation, mesenchymal stem cells

## Abstract

Inflammatory and autophagy-related gene P62 is highly expressed in most human tumor tissues. Herein, we demonstrate that P62 promotes human mesenchymal stem cells’ malignant transformation via the cascade of P62-tumor necrosis factor alpha (TNF-α)-CUDR-CTCF-insulin growth factor II (IGFII)-H-Ras signaling. Mechanistically, we reveal P62 enhances IGFII transcriptional activity through forming IGFII promoter-enhancer chromatin loop and increasing METTL3 occupancy on IGFII 3′ UTR and enhances H-Ras overexpression by harboring inflammation-related factors, e.g., TNFR1, CLYD, EGR1, NFκB, TLR4, and PPARγ. Furthermore, the P62 cooperates with TNF-α to promote malignant transformation of mesenchymal stem cells. These findings, for the first time, provide insight into the positive role that P62 plays in malignant transformation of mesenchymal stem cells and reveal a novel link between P62 and the inflammation factors in mesenchymal stem cells.

## Introduction

Mesenchymal stromal cells (MSCs) are a kind of stromal cell within the tumor microenvironment.^1^ Studies have revealed MSCs tended to directionally migrate toward tumor cells and could mediate stable expression of interleukin-12 (IL-12).^2^ However, the possibility that MSCs have a potential for malignant transformation was raised.

At present, there is no report about the functions of P62 in MSCs. The P62 is a multifunctional adaptor protein that plays an important role at the crossroad between autophagy and cancer.^3^ Recent findings link P62 activity to the extrinsic apoptosis, autophagy, and tumorigenesis.^4^ In particular, interrupting TRB3/P62 interaction produces potent antitumor efficacies against tumor growth and metastasis.^5^ Moreover, altered P62 expression caused NF-E2-related factor 2 (NRF2) activation in cancer stem cells (CSCs)-enriched mammospheres.^6^ Furthermore, P62 is assembled on selective autophagic cargos and is subsequently phosphorylated in an mTORC1-dependent manner.^7^ Moreover, P62 upregulation is commonly observed in human tumors and contributes directly to tumorigenesis.^4^, ^8^ Strikingly, P62 is necessary for Ras to trigger IkappaB kinase (IKK) through the polyubiquitination of tumor necrosis factor receptor (TNFR)-associated factor 6 (TRAF6).^9^

RETRACTED

Transcriptional repressor CTCF, N(6)-methyladenosine (m6A), and inflammation may play a role in MSCs involved in P62. CTCF, also known as 11-zinc finger protein or CCCTC-binding factor, is a transcription factor.^10^, ^11^ CTCF/cohesin-binding sites are frequently mutated in cancer.^12^ CTCF may also play a key role in the pluripotency of cells through the regulation of miR-290 cluster.^13^ m6A methyltransferase METTL3 is an RNA methyltransferase implicated in mRNA biogenesis, decay, and translation control.^14^ Moreover, METTL3 can promote the expression of several crucial oncoproteins, and its high expression enhanced proliferation, survival, and invasion of cancer cells.^15^ Furthermore, specific inhibition of m6A methylation is sufficient to elicit circadian period elongation and RNA processing delay.^16^ Also, genetic inactivation or depletion of METTL3 led to m6A erasure on select target genes.^17^ In particular, the mRNA methylation based on m6A facilitates resolution of naive pluripotency toward differentiation.^18^, ^19^ Inflammation is associated with cancer-prone microenvironment. For example, TNF-α is a pleiotropic cytokine that triggers cell proliferation, cell death, or inflammation.^20^, ^21^ However, cytokine IL-32α suppresses colorectal cancer growth via TNFR1 signaling pathway.^22^

In this study, our aim was to explore the precise mechanism of P62 combined with TNF-α in carcinogenesis, especially the role in the malignant process of mesenchymal stem cells.

## Results

### Malignant Transformation of Mesenchymal Stem Cells in Injured Mouse Liver with Excessive P62

To explore whether inflammation-related gene P62 triggers the malignant transformation of mesenchymal stem cells in the inflammation microenvironment of liver, we first perform liver multiple transfection *in vivo* with pCMV6-AC-GFP, pCMV6-AC-GFP-P62, and pGFP-V-RS-P62 plasmids. Compared with pCMV6-AC-GFP transfected athymic Balb/C mice (severe combined immunodeficiency mice), pCMV6-AC-GFP-P62 multiple transfected mice expressed a fusion protein GFP-P62, and P62 was depleted in pGFP-V-RS-P62 multiple transfected mice (Figure 1A). We selected human-bone-marrow-derived mesenchymal stem cells (HBMMSCs) for experiments according to the schematic diagram (Figure 1B). These HBMMSCs were inoculated into the mouse liver capsule under the B ultrasound guide. The experimental groups included pCMV6-AC-GFP, pCMV6-AC-GFP-P62, pGFP-V-RS-P62, pCMV6-AC-GFP plus carbon tetrachloride (CCL_4_), pCMV6-AC-GFP-P62 plus CCL4, and pGFP-V-RS-P62 plus CCL4. As expected, HBMMSCs were transformed into the tumor in mouse liver with the excessive GFP-P62 plus CCL4 treatment (0.206 ± 0.005 g; n = 8; Figures 1C and 1D), whereas the rest of the groups did not get tumors at all (Figures 1C and 1E). Moreover, these recovered xenografts were poorly differentiated malignant tumors (Figure 1F). Furthermore, human carcino-embryonic antigen (CEA) was expressed in these xenografts (Figure S1A). Taken together, these observations provide evidence that HBMMSCs can cause malignant transformation in injured mouse liver with excessive P62.

RETRACTED

**Figure 1:** Human Mesenchymal Stem Cells Were Subjected to Transformation in Mouse Liver Overexpressing P62 (A) Mouse athymic Balb/C mouse (a severe combined immunodeficiency mouse) liver *in vivo* transfection with pCMV6-AC-GFP, pCMV6-AC-GFP-P62, and pGFP-V-RS-P62 plasmids. The western blotting analysis with anti-P62 in mice liver tissue is shown. β-actin as internal control is shown. (B) The schematic illustrates that mouse mesenchymal stem cells, in which P62 was overexpressed or knocked down, were injected into the athymic Balb/C mouse liver capsule under the B ultrasound guide. Mice were fed with carbon tetrachloride (CCL_4_) for three months. (C) The mice were stratified, the tumors recovered, and xenograft tumor photographed in the six groups as indicated in left. (D) The wet weight of each tumor for each mouse in pCMV6-AC-GFP-P62 plus CCL4 group. (E) The wet weight of each tumor was determined for each mouse. Each value was presented as mean ± SEM; **p < 0.01. (F) A portion of each tumor was fixed in 4% paraformaldehyde and embedded in paraffin for histological H&E staining. The representative analytic results of H&E are shown (100×).

### Excessive P62 Accelerates Malignant Growth of Mesenchymal Stem Cells in Coordination with TNF-α

To investigate whether P62 cooperates with TNF-α to trigger malignant transformation of HBMMSCs, we designed the experimental strategy outlined in Figure 2A. We first constructed HBMMSCs cell lines with stable overexpression or depletion of P62. Four stable cell lines were established by transfecting HBMMSCs with pCMV6-A-GFP (GFP control vector), pCMV6-A-GFP-P62 (P62 expression vector), pGFP-V-RS (RNAi control vector), or pGFP-V-RS-P62(RNAi) (P62 RNAi vector). The P62-overexpressing or knocked down HBMMSCs were then treated with TNF-α or PBS for eight weeks. Then, P62, NF-ƘB, IκBα, and CLYD expression was detected in these transfected cells. As shown in Figure 2B, the level of P62 was increased in P62-overexpressing HBMMSCs and reduced in P62 knockdown HBMMSCs. In HBMMSCs treated with TNF-α, the expression of NFƘB and CLYD was increased in P62-overexpressing HBMMSCs and reduced in P62 knockdown HBMMSCs cells, and the expression of IκBα was decreased in P62-overexpressed HBMMSCs cells and increased in the P62 knockdown. However, in the control group, both P62 overexpression and knockdown did not significantly alter expression of NF-ƘB, CLYD, and IκBα. Next, we examined the growth curves of the HBMMSC lines by the CCK8 assay in the eight groups: pCMV6-AC-GFP+TNF-α; pCMV6-AC-GFP-P62+TNF-α; pGFP-V-RS+TNF-α; and pGFP-V-RS-P62+IL-6, pCMV6-AC-GFP, pCMV6-AC-GFP-P62, pGFP-V-RS, and pGFP-V-RS-P62. As shown in Figure S1B, in TNF-α-treated groups, P62 overexpression significantly increased and P62 knockdown significantly inhibited the growth of HBMMSCs compared to the control cells. However, in the TNF-α-untreated group, this potential role of P62 was fully abrogated. To further address this issue, we detected the S phase cells by bromodeoxyuridine (BrdU) staining. As shown in Figure S1C, in TNF-α-treated groups, P62 overexpression significantly increased (68.9% ± 15.7% versus 32.4% ± 8.2%; p < 0.01) and P62 knockdown significantly inhibited (14.2% ± 2.6% versus 37.8% ± 5.7%; p < 0.01) the BrdU-positive HBMMSCs cells compared to the control cells. However, in TNF-α-untreated groups, either P62 overexpression or knockdown did not significantly alter the rate of BrdU-positive HBMMSCs (34.4% ± 9.1% versus 29.3% ± 6.7% and 26.8% ± 4.2% versus 32.5% ± 5.4%; p > 0.05, respectively).

RETRACTED

**Figure 2:** P62 Overexpression Combined with TNF-α Triggers Malignant Transformation of Human Mesenchymal Stem Cells *In Vitro* and *In Vivo* (A) The schematic illustrates that human mesenchymal stem cells stably transfected with P62 overexpression or knockdown plasmids were transformed into cancer cells that were then treated with TNF-α or control, including groups of pCMV6-AC-GFP (GFP control), pCMV6-AC-GFP-P62 (GFP-P62), pGFP-V-RS (RNAi control), pGFP-V-RS–P62 (P62 RNAi), pCMV6-AC-GFP plus TNF-α, pCMV6-AC-GFP-P62 plus TNF-α, pGFP-V-RS plus TNF-α, and pGFP-V-RS–P62 plus TNF-α. (B) The western blotting analysis with anti-P62, anti-NF-κB, and anti-CLYD in these human mesenchymal stem cells indicated in upper. β-actin and GAPDH as internal control are shown. (C) Cells soft-agar colony formation assay. (D) Cells sphere-formation ability. (E) *In vivo* test in these human mesenchymal stem cells. The mice were stratified, and the tumors were recovered. (F) The wet weight of each tumor was determined for each mouse. Each value was presented as mean ± SEM (Student’s t test). **p < 0.01.

RETRACTED

We further performed soft-agar colony formation assay. As shown in Figure 2C, colony-formation efficiency rate was 54.7% ± 13.8% in the pCMV6-A-GFP-P62 plus TNF-α group, whereas the rest of the groups did not exhibit colony formation (p < 0.01). Similarly, self-renewing sphere-formation rate was 28.8% ± 7.3% in the pCMV6-A-GFP-P62 plus TNF-α group, whereas no sphere formation was observed in the rest of the groups (p < 0.01; Figure 2D). Furthermore, we constructed the stable HBMMSC lines with excessive P62 plus TNFR knockdown. As shown in Figure S2A, TNFR expression was reduced in group of GFP-P62plus pGFP-V-RS-TRFR plus TNF-α. We further performed soft-agar colony formation assay. As shown in Figure S2B, colony-formation efficiency rate was 41.13% ± 8.1% in the pCMV6-A-GFP-P62+ TNF-α group, whereas both the control group and GFP-P62 plus pGFP-V-RS-TNFR plus TNF-α group did not exhibit colony formation (p < 0.01). Similarly, self-renewing sphere-formation rate was 21% ± 4.45% in the pCMV6-A-GFP-P62+ TNF-α group, whereas no sphere formation was observed in the control group or GFP-P62 plus pGFP-V-RS-TRFR plus TNF-α group (p < 0.01; Figure S2C).

To further determine whether P62 plus TNF-α promotes HBMMSC malignant transformation *in vivo* cooperatively, the eight groups of cell lines were injected subcutaneously into the armpit into athymic Balb/C mice. The xenograft tumors were formed only in the P62-overexpressing plus TNF-α-treated HBMMSC groups (0.72 ± 0.151 g; n = 8; compared to control p < 0.01). No tumors were observed in the rest of the groups (Figures 2E and 2F). H&E staining of the xenografts revealed poorly differentiated malignant tumor cells (Figure S3). Moreover, the three groups of cell lines, including GFP-control+TNF-α, GFP-P62+TNF-α, and GFP-P62+pGFP-V-RS-TNFR+TNF-α, were injected subcutaneously into the armpit into athymic Balb/C mice, respectively. The xenograft tumors were formed only in the P62-overexpressing plus TNF-α-treated HBMMSC groups (0.805 ± 0.175 g; n = 6; p < 0.01). No tumors were observed in the control group or GFP-P62 plus pGFP-V-RS-TNFR plus TNF-α group (Figure S2D). Taken together, these observations suggest excessive P62 combined with TNF-α collaboratively triggers malignant transformation and growth of human mesenchymal stem cells.

### P62 Enhances IGFII Transcriptional Activity in the Mesenchymal Stem Cells

To explore whether P62 impacts on insulin growth factor II (IGFII) expression on the level of transcription, we first performed RNA immunoprecipitation (RIP) assay in HBMMSCs. As shown in the Figure 3A, the interplay between CTCF and CUDR was enhanced in P62-overexpressing HBMMSCs and attenuated in P62 knocked down HBMMSCs compared to the corresponding control in HBMMSCs treated with TNF-α. However, the interplay between CTCF and CUDR was not significantly altered either in P62-overexpressing or P62 knocked down HBMMSCs without TNF-α treatment. Furthermore, we carried out chromosome conformation capture (3C)-chromatin immunoprecipitation (ChIP) experiments in TNF-α-treated HBMMCs transfected with pCMV6-AC-GFP, pCMV6-AC-GFP-P62, pGFP-V-RS, and pGFP-V-RS-P62. The IGFII H19 ICR-IGFII DMR2 DNA looping mediated by CTCF was significantly increased in P62-overexpressing HBMMSCs and reduced in P62 knocked down HBMMSCs compared to the corresponding control. Intriguingly, there was more RNA polymerase II into the DNA looping in the P62 excessive HBMMCs and less RNA polymerase II into the DNA looping in the P62 knocked down HBMMCs than in control (Figure 3B). However, after CUDR was knocked down in TNF-α-treated HBMMCs transfected with pCMV6-AC-GFP, pCMV6-AC-GFP-P62, pGFP-V-RS, or pGFP-V-RS-P62, the IGFII H19ICR-IGFII DMR2 DNA looping was rarely produced and less RNA polII entered into the looping in the four groups (Figure 3C). Moreover, IGFII promoter luciferase activity was heightened in the P62-overexpressing HBMMCs and weakened in the P62 knocked down HBMMCs (Figure 3D). Together, these observations suggest P62 boosts the IGFII transcriptional activity dependent on CTCF and long non-coding RNA (lncRNA) CUDR.

RETRACTED

**Figure 3:** P62 Regulates IGFII Transcriptional Activity in the Mesenchymal Stem Cells with TNF-α Treatment (A) RNA immunoprecipitation (RIP) with anti-CTCF followed by RT-PCR with CUDR mRNA primers in the mesenchymal stem cells treated with TNF-α and transfected with pCMV6-AC-GFP (GFP-control), pCMV6-AC-GFP-P62 (GFP-P62), pGFP-V-RS (RNAi control), and pGFP-V-RS–P62 (P62 RNAi). IgG RIP was used as negative control. CUDR RNA as INPUT is shown. (B) Chromosome conformation capture (3C)-chromatin immunoprecipitation (ChIP) with anti-CTCF and anti-RNA polII in the mesenchymal stem cells treated with TNF-α and transfected with pCMV6-AC-GFP, pCMV6-AC-GFP-P62, pGFP-V-RS, and pGFP-V-RS-P62. The PCR analysis is applied for detecting IGFII H19ICR-IGFII DMR2 coupling product using H19ICR and IGFII DMR2 primers. The H19ICR and IGFII DMR2 as INPUT are shown. (C) 3C-ChIP with anti-CTCF and anti-RNA polII in the CUDR knockdown mesenchymal stem cells transfected with pCMV6-AC-GFP, pCMV6-AC-GFP-P62, pGFP-V-RS, and pGFP-V-RS-P62. The PCR analysis is applied for detecting IGFII H19ICR-IGFII DMR2 coupling product using H19ICR and IGFII DMR2 primers. The H19ICR and IGFII DMR2 as INPUT are shown. (D) IGFII promoter luciferase activity assay in in the mesenchymal stem cells treated with TNF-α and transfected with pCMV6-AC-GFP, pCMV6-AC-GFP-P62, pGFP-V-RS, and pGFP-V-RS-P62. Each value was presented as mean ± SEM. **p < 0.01.

RETRACTED

### P62 Exacerbates the METTL3 Occupancy on IGFII mRNA 3′ UTR

We speculated P62 may regulate the METTL3 occupancy on IGFII mRNA. To address this hypothesis, we performed RIP, co-immunoprecipitation (IP), DNA pull-down, super-electrophoretic mobility shift assay (EMSA) (gel-shift) in the TNF-α-treated HBMMSCs transfected with pCMV6-AC-GFP, pCMV6-AC-GFP-P62, pGFP-V-RS, and pGFP-V-RS-P62. As shown in Figure 4A, the interplay between METTL3 and CUDR was increased in P62-overexpressing HBMMSCs and attenuated in P62 knocked down HBMMSCs. However, in HBMMSCs without TNF-α treatment, the interplay between METTL3 and CUDR did not change either P62-overexpressing or P62 knockdown. Furthermore, the interplay between METTL3 and CTCF was increased in P62-overexpressing HBMMSCs and attenuated in P62 knocked down HBMMSCs compared to the corresponding controls. However, when the CUDR was knocked down, the interplay between METTL3 and CTCF was not changed in these cells (Figure 4B). Moreover, CUDR RNA pull-down assay showed that the interplay among CTCF, METTL3, and CUDR was increased in P62-overexpressing HBMMSCs and attenuated in P62 knocked down HBMMSCs compared to the corresponding controls (Figure 4C). Furthermore, METTL3 expression was increased in P62-overexpressing plus TNF-α-treated HBMMSCs as well as decreased in P62 knocked down plus TNF-α-treated HBMMSCs compared to the corresponding controls (Figure 4D). In addition, the FTO expression did not alter in these cell lines (Figure 4D). Interestingly, RIP analysis shows that the interplay between METTL3 and IGFII mRNA was increased in P62-overexpressing HBMMSCs and attenuated in P62 knocked down HBMMSCs compared to the corresponding control. However, in HBMMSCs without the TNF-α treatment or CUDR knocked down, the interplay between METTL3 and IGFII mRNA was not significantly altered in cells with P62 overexpression or P62 knockdown (Figure 4E). Furthermore, the super-EMSA showed that the interplay between METTL3 and IGFII mRNA probe was increased in P62-overexpressing HBMMSCs and attenuated in P62 knocked down HBMMSCs compared to the corresponding control (Figure 4F). Then, we quantified the super-METTL3 bands in each lane in Figure 4F by calculating the gray density value of super-METTL3 bands. The results showed that the interplay between METTL3 and IGFII mRNA probe was increased in P62-overexpressing HBMMSCs (1.89 ± 0.34 versus 5.52 ± 0.53; n = 3; p = 0.009 < 0.01) and attenuated in P62 knocked down HBMMSCs compared to the corresponding control (168 ± 0.29 versus 0.31 ± 0.06; n = 3; p = 0.0075 < 0.01; Figure 4G). These observations suggest that P62 enhances the METTL3 occupancy on IGFII mRNA dependent on lncRNA CUDR and insulator CTCF in the inflammatory environment.

RETRACTED

**Figure 4:** The P62 Enhanced the METTL3 Occupancy on IGFII mRNA 3′ UTR in the Mesenchymal Stem Cells with TNF-α Treatment (A) RIP with anti-METTL3 followed by RT-PCR with CUDR mRNA primers in the mesenchymal stem cells treated with TNF-α and transfected with pCMV6-AC-GFP (GFP-control), pCMV6-AC-GFP-P62 (GFP-P62), pGFP-V-RS (RNAi control), and pGFP-V-RS-P62 (P62 RNAi). IgG RIP as negative control is shown. CUDR mRNA as INPUT is shown. (B) Anti-CTCF co-IP followed by western blotting with anti-METTL3 primers in the mesenchymal stem cells treated with TNF-α or CUDR knockdown and transfected with pCMV6-AC-GFP, pCMV6-AC-GFP-P62, pGFP-V-RS, and pGFP-V-RS-P62. IgG IP as negative control is shown. INPUT refers to western blotting with anti-CTCF. (C) Biotin-CUDR cDNA pull-down followed by western blotting with anti-MELLT3 and anti-CTCF primers in the mesenchymal stem cells treated with TNF-α and transfected with pCMV6-AC-GFP, pCMV6-AC-GFP-P62, pGFP-V-RS, and pGFP-V-RS-P62. Biotin as INPUT and histone as internal control are shown. (D) Western blotting with anti-METTL3 and anti-FTO in the mesenchymal stem cells treated with TNF-α and transfected with pCMV6-AC-GFP, pCMV6-AC-GFP-P62, pGFP-V-RS, and pGFP-V-RS-P62. β-actin as internal control is shown. (E) RIP with anti-METTL3 followed by RT-PCR with IGFII mRNA primers in the mesenchymal stem cells treated with TNF-α or CUDR knockdown and transfected with pCMV6-AC-GFP, pCMV6-AC-GFP-P62, pGFP-V-RS, and pGFP-V-RS-P62. IgG RIP as negative control is shown. IGFII mRNA as INPUT is shown. (F) Super-EMSA (gel-shift) with biotin-IGFII cRNA probe and anti-METTL3 antibody in the mesenchymal stem cells treated with TNF-α and transfected with pCMV6-AC-GFP, pCMV6-AC-GFP-P62, pGFP-V-RS, and pGFP-V-RS-P62. The intensity of the band was examined by western blotting with anti-biotin. (G) The super-METTL3 bands were quantified by calculating the band gray density value (n = 3). Each value was presented as mean ± SEM. **p < 0.01.

### P62 Enhances IGFII Expression

To confirm whether P62 increases the IGFII expression in the mesenchymal stem cells, we first examined the influence of P62 on methylation of IGFII mRNA. RIP with anti-N6Ame results showed that the methylation of IGFII mRNA was increased in P62 -overexpressing HBMMSCs treated with TNF-α and reduced in P62 knocked down HBMMSCs treated with TNF-α compared to corresponding control (Figure 5A). Super-EMSA (gel-shift) with biotin-IGFII RNA probe and anti-N6Ame antibody results showed that the methylation of IGFII mRNA (N6Ame-bound IGFII mRNA) was increased in P62-overexpressing HBMMSCs treated with TNF-α and reduced in P62 knocked down HBMMSCs treated with TNF-α compared to corresponding control (Figure 5B). IGFII mRNA biotin-probe pull-down followed by the run-on assay with anti-N6Ame (Figure 5Ca) and IGFII mRNA biotin-probe pull-down followed northern-western blotting assay with anti-N6Ame (Figure 5Cb) showed that the methylation of IGFII mRNA was increased in P62-overexpressing HBMMSCs treated with TNF-α and reduced in P62 knocked down HBMMSCs treated with TNF-α compared to the corresponding controls. Moreover, IGFII promoter luciferase activity assay showed that miR122 targeted for IGFII mRNA 3′ UTR and P62 raised the IGFII mRNA 3′ UTR activity. In particular, P62 fully abolished the miR122 action (Figure 5Da). miR122 inhibited IGFII expression, and P62 increased the IGFII expression. Moreover, P62 fully abolished this miR122 effect (Figure 5Db). Strikingly, both RT-PCR (Figure 5E) and western blotting (Figure 5F) results showed that IGFII was increased in P62-overexpressing HBMMSCs treated with TNF-α and reduced in P62 knocked down HBMMSCs treated with TNF-α compared to the corresponding controls. In particular, phosphorylated IGFII (pIGFII) was increased in P62-overexpressing HBMMSCs treated with TNF-α and reduced in P62 knocked down HBMMSCs treated with TNF-α compared to the corresponding controls (Figure 5F). Together, these observations suggest that P62 increased the methylation on IGFII mRNA 3′ UTR and the expression of IGFII in the mesenchymal stem cells under inflammatory condition.

RETRACTED

**Figure 5:** The P62 Promotes the Methylation on IGFII mRNA and Its Expression in the TNF-α-Treated Mesenchymal Stem Cells Transfected with pCMV6-AC-GFP (GFP-Control), pCMV6-AC-GFP-P62 (GFP-P62), pGFP-V-RS (RNAi Control), or pGFP-V-RS-P62 (P62 RNAi) (A) RIP with anti-N6Ame followed by RT-PCR with IFGII mRNA primers. IgG RIP as negative control is shown. IGFII mRNA was used as INPUT. (B) Super-EMSA (gel-shift) with biotin-IGFII cRNA probe and anti-N6Ame antibody. The intensity of the band was examined by western blotting with anti-biotin. (C) (a) IGFII rRNA biotin-probe pull-down followed run on assay with anti-N6Ame. Biotin as internal control is shown. (b) IGFII rRNA biotin-probe pull-down followed northern-western blotting assay with anti-N6Ame is shown. Histone as internal control is shown. (D) (a) Western blotting with anti-IGFII in the TNF-α-treated mesenchymal stem cells transfected with pCMV-mir (control), pCMV-miR122, pCMV6-AC-GFP-P62 (GFP-P62), or pCMV-miR122 plus pCMV6-AC-GFP-P62 (GFP-P62). β-actin was used as an internal control. (b) The IGFII 3′ UTR luciferase activity assay in the TNF-α-treated mesenchymal stem cells transfected with pCMV-mir, pCMV-miR122, pCMV6-AC-GFP-P62, and pCMV-miR122 plus pCMV6-AC-GFP-P62 is shown. (E) RT-PCR with IGFII mRNA primers in the TNF-α-treated mesenchymal stem cells transfected with pCMV6-AC-GFP (GFP-control), pCMV6-AC-GFP-P62 (GFP-P62), pGFP-V-RS (RNAi control), or pGFP-V-RS-P62 (P62 RNAi). β-actin served as internal control. (F) Western blotting with anti-IGFII and anti-pIGFII in the TNF-α-treated mesenchymal stem cells transfected with pCMV6-AC-GFP, pCMV6-AC-GFP-P62, pGFP-V-RS, and pGFP-V-RS-P62. β-actin was used as an internal control. **p < 0.01.

RETRACTED

### P62 Promotes the Expression and Phosphorylation of H-Ras via IGFII

Given that P62 increased the IGFII expression in the mesenchymal stem cells, it was reasonable to consider whether P62 enhanced H-Ras expression dependent on IGFII. We first performed anti-IGFII co-IP assay in the TNFα-treated HBMMSCs. As shown in Figure 6A, the interplay between IGFII and P62, TNFR1, CLYD, EGR1, NFκB, TLR4, and PPARγ was increased in P62-overexpressing HBMMSCs and reduced in P62 knocked down HBMMSCs compared to corresponding control. ChIP results showed that the occupancy ability of IGFII, P62, TNFR1, CLYD, NFκB, TLR4, or PPARγ on H-Ras promoter DNA region was enhanced in P62-overexpressing HBMMSCs and attenuated in P62 knocked down HBMMSCs compared to the corresponding controls (Figure 6B). Furthermore, H-Ras promoter luciferase activity was increased in P62-overexpressing HBMMSCs and reduced in P62 knocked down HBMMSCs compared to corresponding control (Figure 6C). RT-PCR results showed that H-Ras mRNA was increased in P62-overexpressing HBMMSCs and decreased in P62 knocked down HBMMSCs compared to the corresponding controls (Figure 6D). Moreover, the expression and phosphorylation of H-Ras was increased in P62-overexpressing HBMMSCs and decreased in P62 knocked down HBMMSCs compared to corresponding control (Figure 6E). Although the expression and phosphorylation of H-Ras were increased in P62-overexpressing HBMMSCs, IGFII knockdown fully abrogated the action of P62 (Figure S4). Collectively, P62 enhanced H-Ras expression and its phosphorylation in the human mesenchymal stem cells in an inflammatory environment.

**Figure 6:** IFGII Induced Overexpression of H-Ras in the Mesenchymal Stem Cells (A) Anti-IGFII co- IP followed by western blotting with anti-P62,anti-TNFR1, anti-CLYD, anti-EGR1, anti-NFκB, anti-TLR4, and anti-PPARγ in the TNF-α-treated mesenchymal stem cells transfected with pCMV6-AC-GFP, pCMV6-AC-GFP-P62, pGFP-V-RS, pGFP-V-RS-P62, and IgG IP as negative control. INPUT refers to western blotting with anti-IGFII. (B) CHIP with anti-IGFII, anti-P62, anti-TNFR1, anti-CLYD, anti-NFκB, or anti-PPARγ followed by PCR with H-Ras promoter primer in the TNF-α-treated mesenchymal stem cells transfected with pCMV6-AC-GFP (GFP-control), pCMV6-AC-GFP-P62 (GFP-P62), pGFP-V-RS (RNAi control), and pGFP-V-RS-P62 (P62 RNAi). IgG CHIP was used as negative control. H-Ras promoter as INPUT is shown. (C) The H-Ras promoter luciferase activity assay in the TNF-α-treated mesenchymal stem cells transfected with pCMV6-AC-GFP (GFP-control), pCMV6-AC-GFP-P62 (GFP-P62), pGFP-V-RS (RNAi control), or pGFP-V-RS-P62 (P62 RNAi). (D) RT-PCR with H-Ras primers in the TNF-α-treated mesenchymal stem cells transfected with pCMV6-AC-GFP (GFP-control), pCMV6-AC-GFP-P62 (GFP-P62), pGFP-V-RS (RNAi control), and pGFP-V-RS-P62 (P62 RNAi), respectively. β-actin as internal control is shown. (E) Western blotting with anti-H-Ras and anti-pH-Ras in the TNF-α-treated mesenchymal stem cells transfected with pCMV6-AC-GFP (GFP-control), pCMV6- AC-GFP-P62 (GFP-P62), pGFP-V-RS (RNAi control), and pGFP-V-RS-P62 (P62 RNAi), respectively. β-actin was used as an internal control. **p < 0.01.

RETRACTED

### The Activated H-Ras Regulates Gene Expression in the Human Mesenchymal Stem Cells

In the light of H-Ras overexpression in P62-transfected plus TNF-α-treated human mesenchymal stem cells, it was reasonable to consider whether H-Ras was activated and the activated H-Ras induced modification and/or abnormal expression of specific genes. At first, we performed glutathione S-transferase (GST) pull-down using GST-Raf1-RBD. As shown in Figure 7A, P62 overexpression enhanced and P62 knockdown reduced the activated H-Ras activity in the TNF-α-treated mesenchymal stem cells. Furthermore, the phosphorylation of Raf, MEKK1, ERK, MEKK4, MEK, Jak, EIK, P38, PI3K, mTOR, and AKT were increased in P62-overexpressing plus TNF-α-treated mesenchymal stem cells and decreased in P62 knockdown plus TNF-α-treated mesenchymal stem cells (Figure 7B). Together, these observations suggest that P62 combined with TNF-α promoted H-Ras activation and the activated H-Ras induced certain gene abnormal phosphorylation modification in the human mesenchymal stem cells.

**Figure 7:** The Activated H-Ras Induced Some Gene Abnormal Expression of Specific Genes in the P62-Overexpressing or Knockdown Mesenchymal Stem Cells Treated with TNF-α (A) GST pull-down using GST-Raf1-RBD system followed by western blotting anti-GTP Ras in the mesenchymal stem cells transfected with pCMV6-AC-GFP (GFP-control), pCMV6-AC-GFP-P62 (GFP-P62), pGFP-V-RS (RNAi control), and pGFP-V-RS-P62 (P62 RNAi). INPUT refers to western blotting with anti-H-Ras. (B) Western blotting with anti-pRaf, anti-Raf, anti-pMEKK1, anti-MEKK1, anti-pERK, anti-ERK, anti-pMEKK4, anti-MEKK4, anti-pMEK, anti-MEK, anti-pJak, anti-Jak, anti-pEIK, anti-EIK, anti-P38, anti-pPI3K, anti-PI3K, anti-pmTOR, or anti-pAKT in the mesenchymal stem cells transfected with pCMV6-AC-GFP (GFP-control), pCMV6-AC-GFP-P62 (GFP-P62), pGFP-V-RS (RNAi control), and pGFP-V-RS-P62 (P62 RNAi). β-actin served as an internal control.

RETRACTED

### Depletion of H-Ras Abrogated the Synergetic Oncogenic Function of the P62 plus TNF-α

To further demonstrate whether the cooperative effect of P62 with TNF-α is through the H-Ras, we performed the rescue experiment. We first constructed the stable HBMMSC lines by transfection and treated with pCMV6-AC-GFP-P62, pCMV6-AC-GFP-P62 plus pcDNA3.1-H-Ras, pCMV6-AC-GFP-P62 plus TNF-α, and pCMV6-AC-GFP-P62 plus TNF-α plus pGFP-V-RS-H-Ras. As shown in Figure 8A, we successfully constructed four groups of cell lines, including P62, P62 plus H-Ras, P62 plus TNF-α, and P62 plus TNF-α plus H-Ras knockdown group. P62 was overexpressed in all four groups, and H-Ras was overexpressed in pCMV6-AC-GFP-P62 plus pcDNA3.1-H-Ras and pCMV6-AC-GFP-P62 plus TNF-α and was knocked down in P62 plus TNF-α plus H-Ras knockdown. Cell growth assay showed more rapid growth in P62 plus TNF-α, and there was no significant difference among the rest of the groups (Figure 8B). Intriguingly, the action of P62 plus TNF-α was fully abrogated after H-Ras was knocked down in the transfected HBMMSCs. We further performed soft-agar colony formation assay. As shown in Figure 8C, colony-formation efficiency rate was 56.81% ± 12.61% in the P62 plus TNF-α group, whereas the rest of the groups did not exhibit colony formation. The four groups of cell lines were injected subcutaneously in the armpit of athymic Balb/C mice. As shown in Figures 8Da and 8Db, only the P62 plus TNF-α HBMMSCs produced xenograft tumors (0.974 ± 0.180 g; n = 7), whereas no tumor formation was observed in the three groups. Furthermore, pathological examination (H&E staining) of the xenografts revealed poorly differentiated tumor cells (Figure S5).

**Figure 8:** The Rescued Experiment of Carcinogenesis Effect of the P62 in TNF-α-Treated Mesenchymal Stem Cells Transfected with pCMV6-AC-P62 (GFP-P62), pCMV6-AC-GFP-P62 (GFP-P62) plus pcDNA3.1-H-Ras (Ras), pCMV6-AC-P62 (GFP-P62) plus TNF-α, and pCMV6-AC-P62 (GFP-P62) plus TNF-α plus pGFP-V-RS-H-Ras (Rasi) (A) Western blotting analysis with anti-P62 and anti-H-Ras in mesenchymal stem cells. β-actin served as internal control. (B) Cells growth assay using CCK8. Each value was presented as mean ± SEM. (C) Cells soft-agar colony formation assay. (D) Tumorigenesis test *in vivo* in these mesenchymal stem cells. (a) The mice were stratified, and the tumors were recovered. (b) The wet weight of each tumor was determined for each mouse. Each value was presented as mean ± SEM. **p < 0.01; *p < 0.05.

RETRACTED

Furthermore, we constructed the stable HBMMSC lines with excessive P62 plus IGFII knockdown. As shown in Figure S4, IGFII expression was reduced in group of GFP-P62 plus pGFP-V-RS-IGFII plus TNF-α. As shown in Figure S6A, P62 overexpression plus TNF-α significantly increased compared to the control cells. However, in the GFP-P62 plus pGFP-V-RS-IGFII plus TNF-α group, this potential role of P62 was fully abrogated. We further performed soft-agar colony formation assay. As shown in Figure S6B, colony-formation efficiency rate was 33.67% ± 6.54% in the pCMV6-A-GFP-P62+ TNF-α group, whereas both the control group and GFP-P62 plus pGFP-V-RS-IGFII plus TNF-α group did not exhibit colony formation (p < 0.01). Similarly, self-renewing sphere-formation rate was 19.97% ± 4.87% in the pCMV6-A-GFP-P62+ TNF-α group, whereas no sphere formation was observed in the control group or GFP-P62 plus pGFP-V-RS-IGFII plus TNF-α group (p < 0.01; Figure S6C).The three groups of cell lines, including GFP-control+TNF-α, GFP-P62+TNF-α, GFP-P62+pGFP-V-RS-IGFII+TNF-α, were injected subcutaneously into the armpit into athymic Balb/C mice, respectively. The xenograft tumors were formed only in the P62-overexpressing plus TNF-α-treated HBMMSCs groups (0.922 ± 0.219 g; n = 6; compared to control p < 0.01). No tumors were observed in the control group or GFP-P62 plus pGFP-V-RS-IGFII plus TNF-α group (Figure S6D).

Furthermore, we prepared the P62 mutant plasmid pCMV6-A-GFP-P62(W338A) and constructed the stable HBMMSC lines with excessive P62 or excessive mutant P62(W338A). As shown in Figure S7A, both GFP-P62 and GFP-P62(W338A) were increased in group of pCMV6-A-GFP-P62 and pCMV6-A-GFP-P62(W338A) compared to pCMV6-AC-GFP control group. The expression of Ras was also significantly increased in pCMV6-AC-GFP-P62 plus TNF-α group compared to the pCMV6-AC-GFP control group. However, in the pCMV6-AC-GFP-P62(W338A) plus TNF-α group, this potential role was fully abrogated. We further performed soft-agar colony formation assay. As shown in Figure S7B, colony-formation efficiency rate was 37.37% ± 8.80% in the pCMV6-A-GFP-P62 plus TNF-α group, whereas both the control group and pCMV6-A-GFP-P62(W338A) plus TNF-α group did not exhibit colony formation (p < 0.01). Similarly, self-renewing sphere-formation rate was 22.2% ± 5.29% in the pCMV6-A-GFP-P62 plus TNF-α group, whereas no sphere formation was observed in the pCMV6-AC-GFP group and pCMV6-A-GFP-P62(W338A) plus TNF-α group (p < 0.01; Figure S7C).

RETRACTED

Taken together, the overexpression of P62 combined with TNF-α resulted in the malignant transformation of HBMMSCs, but the oncogenic activity was fully abrogated by H-Ras depletion or IGFII depletion. Moreover, mutant P62 (W338A) lacks the functions of wild P62 in human mesenchymal stem cells.

## Discussion

Multifunctional scaffold protein P62 is well known as an autophagy marker protein and provides crosstalk for important signaling pathways, including NF-κB signaling. In this study, we demonstrate that P62 promotes malignant differentiation of human mesenchymal stem cells via cascade of P62-TNF-α-CUDR-CTCF-IGFII-H-Ras signaling (Figure 9). To our knowledge, this is the first report demonstrating that P62 cooperates with TNF-α to promote the malignant transformation of mesenchymal stem cells. Obviously, this is a novel linkage of P62-TNF-α-CUDR-CTCF-IGFII-H-Ras signaling to tumorigenesis.

**Figure 9:** The Schematic Illustrates a Model of Malignant Transformation of Human Mesenchymal Stem Cells via P62-TNF-α-CUDR-CTCF-IGFII-H-Ras Axis Mediated by Long Noncoding RNA CUDR P62 enhances IGFII transcriptional activity through forming IGFII promoter-enhancer chromatin loop recruiting RNA polII and increasing METTL3 occupancy on IGFII mRNA 3′UTR, which promotes the methylation of IGFII mRNA in mesenchymal stem cells. The excessive IGFII induces the H-Ras overexpression by harboring more inflammation-related factors, e.g., P62, TNFR1, CLYD, EGR1, NFκB, TLR4, and PPARγ onto the H-Ras promoter region. Subsequently, the excessive H-Ras was activated to induce abnormal expression of gene, e.g., Raf, MEKK1, ERK, MEKK4, MEK, Jak, EIK, P38, PI3K, mTOM, and AKT, in the mesenchymal stem cells. Thereby, P62 cooperates with TNF-α to promote mesenchymal stem cells’ malignant transformation.

It is worth mentioning that P62 plus TNF-α plays an important role in the malignant transformation of mesenchymal stem cells. In this report, we focused mainly on how P62 functions under the inflammatory environment. To date, accumulating evidence indicates that P62 exerts a carcinogenic effect. The P62 knockdown coordinates a series of antiproliferative responses and may facilitate dedifferentiation of mature hepatocytes into nestin-positive progenitor-like cells.^23^, ^24^ Herein, our results showed that P62 cooperates with TNF-α to promote the malignant transformation of mesenchymal stem cells. The involvement of promotion of the malignant transformation of mesenchymal stem cells is supported by results from two parallel sets of experiments: (1) P62 triggers mesenchymal stem cells’ malignant transformation in injury inflammatory mouse liver and (2) excessive P62 cooperates with TNF-α to accelerate mesenchymal stem cells’ malignant growth *in vitro* and *in vivo.* According to the aforementioned findings and reports, it is thus clear that P62 has a strong carcinogenic ability under inflammatory condition.

RETRACTED

It has been confirmed that IGFII is closely associated with hepatocarcinogenesis. Activation of IGF or insulin signaling preserves the survival of cancer cells under special stress.^25^, ^26^ In this report, we have shown that P62 plus TNF-α promotes IGFII expression and phosphorylation. This assertion that P62 enhances IGFII transcriptional activity in the mesenchymal stem cells is based on several observations. (1) The interplay between CTCF and CUDR was enhanced in P62-overexpressing HBMMSCs treated with TNF-α. (2) The IGFII H19 ICR-IGFII DMR2 DNA looping facilitated through CTCF was increased in P62-overexpressing HBMMSCs. (3) IGFII promoter luciferase activity was enhanced in the P62-overexpressing HBMMCs. (4) P62 boosts the IGFII transcriptional activity through insulator CTCF under the control of CUDR. This assertion that P62 enhanced the METTL3 occupancy on IGFII mRNA using long noncoding RNA CUDR and insulator CTCF in the inflammatory environment is based on several observations. (1) The interplay between METTL3 and CUDR was increased in P62-overexpressing HBMMSCs treated with the TNF-α. (2) The interplay between METTL3 and CTCF was increased in P62-overexpressing HBMMSCs. (3) The interaction among CTCF, METTL3, and CUDR was increased in P62-overexpressing HBMMSCs. (4) The interplay between METTL3 and IGFII mRNA was increased in P62-overexpressing HBMMSCs. This assertion that P62 increased the methylation on IGFII mRNA 3′ UTR and its expression is based on several observations. (1) The methylation of IGFII mRNA was increased in P62-overexpressing HBMMSCs treated with TNF-α. (2) The methylation of IGFII mRNA (N6Ame-bound IGF mRNA) was increased in P62-overexpressing HBMMSCs treated with TNF-α. (3) The methylation of IGFII mRNA was increased in P62-overexpressing HBMMSCs treated with TNF-α. (4) miR122 inhibited IGFII expression and P62 increased the IGFII expression; thus, P62 abolished the miR122 effect. (5) IGFII mRNA was increased in P62-overexpressing HBMMSCs treated with TNF-α.

There is plenty of evidence that H-Ras is an oncogene,^27^, ^28^, ^29^ and it is well known that Ras promotes tumorigenesis.^30^, ^31^ Furthermore, K-ras mutation is related to tumorigenesis and metastatisis.^30^, ^35^ In this study, we discovered that P62 enhanced the H-Ras expression and phosphorylation through IGFII in the human mesenchymal stem cells. This assertion is based on several observations. (1) The interplay between IGFII and P62, TNFR1, CLYD, EGR1, NFκB, TLR4, and PPARγ was increased in P62-overexpressing HBMMSCs. (2) The binding of IGFII, P62, TNFR1, CLYD, EGR1, NFκB, TLR4, and PPARγ on H-Ras promoter DNA region was enhanced in P62-overexpressing HBMMSCs. (3) H-Ras promoter luciferase activity was increased in P62-overexpressing HBMMSCs. (4) H-Ras mRNA was increased in P62-overexpressing HBMMSCs. (5) H-Ras expression and its phosphorylation was increased in P62-overexpressing HBMMSCs. This assertion that P62 cooperates with TNF-α to promote H-Ras activation and the activated H-Ras alters gene expression and modification in the human mesenchymal stem cells is based on several observations. (1) P62 overexpression enhanced and P62 knockdown reduced the activated H-Ras form GTP-Ras in the TNF-α-treated mesenchymal stem cells. (2) The phosphorylation of Raf, MEKK1, ERK, MEKK4, MEK, Jak, EIK, P38, PI3K, mTOR, and AKT was increased in P62-overexpressing and TNF-α-treated mesenchymal stem cells. In addition, Akt/mTOR pathway plays a role in tumorigenesis.^32^, ^33^ Our results suggest P62 may be associated with Akt/mTOR pathway in tumorigenesis.

RETRACTED

Although increase in H-Ras may partly contribute to P62 plus TNF-α-mediated promotion of mesenchymal stem cells’ malignant transformation, our findings in this study provide novel evidence for an active role of H-Ras promotion of mesenchymal stem cells’ malignant transformation. This assertion is based on several observations: H-Ras knockdown abrogated the synergetic oncogenic function of the P62 plus TNF-α in mesenchymal stem cells. The action of P62 plus TNF-α was fully abrogated after H-Ras was knocked down in the transfected HBMMSCs, including cell growth, soft-agar colony formation ability, and xenograft tumors formation. It is evident that activation of H-Ras may play an important role in the malignant transformation of mesenchymal stem cells. Our findings in this study provide novel evidence for an active role of P62 plus TNF-α promotion of mesenchymal stem cells malignant transformation.

Our present approaches provided an unequivocal evidence for critical oncogenic roles of P62 plus TNF-α in mesenchymal stem cells’ malignant transformation and supported the notion that P62 plus TNF-α may be an alternative bona fide promoting factor of carcinoma. We presented three novel mechanisms for P62 plus TNF-α role in the malignant transformation of mesenchymal stem cells. First, P62 intensifies IGFII transcriptional activity through forming IGFII promoter-enhancer chromatin loop recruiting RNApolII and increasing METTL3 occupancy on IGFII 3′ UTR mRNA. Second, the excessive IFGII induced the H-Ras overexpression by harboring more inflammation-related factors, e.g., TNFR1, CLYD, EGR1, NFκB, TLR4, and PPARγ onto the H-Ras promoter region. And third, excessive H-Ras was activated and induced abnormal expression of genes, including Raf, MEKK1, ERK, MEKK4, MEK, Jak, EIK, P38, PI3K, mTOR, and AKT in the mesenchymal stem cells. On the basis of these mechanisms, P62 plus TNF-α exerts a tumorigenic function through P62-TNF-α-CUDR-CTCF-IGFII-H-Ras cascade signaling pathway in mesenchymal stem cells. In the future, the important role P62-TNF-α-CUDR-CTCF-IGFII-H-Ras axis might play in carcinogenesis and progression remains to be elucidated. However, we do not fully understand the mechanism of P62 plus TNF-α. Some of the outstanding questions include: how do P62 plus TNF-α control IGFII change and modification? How do P62 plus TNF-α regulate H-Ras expression? What are the recruitment factors and partners of P62 plus TNF-α during the regulation and control of several genes? What is the clinic significance of P62 plus TNF-α? Our present findings open the possibility that targeting P62 plus TNF-α might prove to be an alternative therapeutic strategy. For example, baculovirus-mediated microRNA (miRNA) regulation may be used to suppress hepatocellular tumorigenicity and metastasis.^34^ These findings provide insight into the positive role P62 plays in mesenchymal stem cells’ malignant transformation through the cascade of P62-TNF-α-CUDR-CTCF-IGFII-RAS signaling under the inflammation condition and reveal a novel link between P62 and the inflammation factors in mesenchymal stem cells.

RETRACTED

## Materials and Methods

### Cell Lines and Plasmids

Normal HBMMSCs were purchased from ATCC (ATCC PCS-500-012; ATCC, Manassas, VA). HBMMSCs were maintained in DMEM supplemented with 10% heat-inactivated fetal bovine serum (Gibco) in a humidified atmosphere of 5% CO_2_ incubator at 37°C. Plasmid pGFP-V-RS, pCMV6-AC-GFP, pMiR-Target, and pCMV-miR were purchased from Origene (Rockville, MD 20850, USA). pCMV-miR122, pGFP-V-RS-P62, pGFP-V-RS-CUDR, pGFP-V-RS-H-Ras, pCMV6-AC-GFP-P62, and pMiR-target-IGFII 3′ UTR were prepared by the authors. The short hairpin RNA (shRNA) includes as follows: CUDR short hairpin RNA (shRNA): 5′-TTCAGACTCAGCCCACTTGCACCCAAGTG-3′; P62 shRNA: 5′- GGCTTCCAGGCGCACTACCGCGATGAGGA-3′; Ras shRNA: 5′- CCAGAACCACTTTGTGGACGAGTATGATC-3′.

### Mouse Liver *In Vivo* Transfection and Liver Transplantation of the HBMMSCs

Systemic administration of athymic Balb/C mouse (a severe combined immunodeficiency mouse) using liver *in vivo* transfection reagent (Altogen Biosystems, Las Vegas, NV 89107, USA) conjugated with plasmid DNA (pCMV6-AC-GFP, pCMV6-AC-GFP-P62, and pGFP-V-RS-P62) was performed according to manufacturer’s instructions. Viable HBMMSCs (10^8^ cells/mouse) were inoculated into liver of athymic Balb/C mouse. The Balb/C mice were observed three months and then sacrificed and the tumors recovered. The wet weight of each tumor was determined for each mouse. A portion of each tumor was fixed in 4% paraformaldehyde and embedded in paraffin for histological H&E staining.

RETRACTED

### RT-PCR

Total RNA was purified using Trizol (Invitrogen) according to manufacturer’s instructions. PCR analysis was performed under the special conditions. β-actin was used as an internal control.

### Western Blotting

Cellular proteins were separated on a 10% SDS-PAGE and transferred onto a nitrocellulose membrane, blocked in 10% dry milk-TBST for 1 hr at 37°C. Following three washes in Tris-HCl (pH 7.5) with 0.1% Tween 20, the blots were incubated with antibodies overnight at 4°C. Following three washes, membranes were then incubated with secondary antibody. Standard western blotting procedures were used with the following antibodies: mouse monoclonal anti-P62 (1:1,000); mouse monoclonal anti-NFƘB (1:1,000); rabbit polyclonal anti-CLYD (1:1,000); mouse monoclonal anti-CTCF (1:1,000); rabbit polyclonal anti-RNA polII (1:1,000); rabbit polyclonal anti- IGFII (1:1,000); mouse monoclonal anti-METTL3 (1:1,000); mouse monoclonal anti-FTO (1:1,000); mouse monoclonal anti-TNFR1 (1:500); mouse monoclonal anti-EGR1 (1:1,000); mouse monoclonal anti-TLR4 (1:1,000); rabbit polyclonal anti-PPARγ (1:500); rabbit polyclonal anti-pRaf (1:1,000); rabbit polyclonal anti-Raf (1:1,000); rabbit polyclonal anti-pMEKK1 (1:200); anti-MEKK1 (1:200); rabbit polyclonal anti-pERK (1:1,000); rabbit polyclonal anti-ERK (1:1,000); rabbit polyclonal anti-pMEKK4 (1:500); rabbit polyclonal anti-MEKK4 (1:500); rabbit polyclonal anti-pMEK (1:1,000); rabbit polyclonal anti-MEK (1:500); rabbit polyclonal anti-pJak (1:500); rabbit polyclonal anti-Jak (1:1,000); rabbit polyclonal anti-pEIK (1:1,000); rabbit polyclonal anti-EIK (1:1,000); mouse monoclonal anti-P38 (1:1,000); mouse monoclonal anti-pPI3K (1:500); mouse monoclonal anti-PI3K (1:1,000); mouse monoclonal anti-pmTOM (1:1,000); mouse monoclonal anti-mTOR (1:1,000); rabbit polyclonal anti-pAKT (1:500); and mouse monoclonal anti-β-actin (1:2,000) were purchased from Santa Cruz Biotechnology, Cell Signaling Technology, and Abcam. IRDye 680LT/IRDye 800CW secondary antibodies (1:50,000) were purchased from LI-COR Scientific Company.

### Co-IP

Protein was pre-cleared with protein G/A-plus agarose beads (Santa Cruz Biotechnology, CA) for 1 hr at 4°C, and the supernatant was obtained after centrifugation (3,000 rpm) at 4°C. Pre-cleared homogenates (supernatant) were incubated with antibodies and/or normal mouse/rabbit immunoglobulin G (IgG) with rotation for 4 hr at 4°C. The immunoprecipitates were incubated with protein G/A-plus agarose beads by rotation overnight at 4°C and then centrifuged at 3,000 rpm for 5 min at 4°C. The precipitates were washed five times for 10 min with beads wash solution and resuspended in loading buffer. Western blotting was performed with related antibodies.

RETRACTED

### ChIP Assay

Cells were cross-linked with 1% (v/v) formaldehyde for 10 min at room temperature and stopped with 125 mM glycine for 5 min. Cross-linked cells were washed with PBS, resuspended in lysis buffer, and sonicated for 8–10 min in a SONICS VibraCell. Chromatin extracts were pre-cleared with protein-A/G-Sepharose beads and immunoprecipitated with antibodies on protein-A/G-Sepharose beads. After washing, elution, and de-cross-linking, the ChIP DNA was detected by PCR.

### Super-EMSA (Gel-Shift)

Cells were washed and scraped in ice-cold PBS to prepare nuclei for electrophoretic gel mobility shift assay with the use of the gel shift assay system modified according to the manufacturer’s instructions (Promega).

### GST Pull-Down

GST pull-down was performed using GST-Raf1-RBD system (Thermo Scientific Pierce) followed by western blotting with anti-GTP Ras in the mesenchymal stem cells transfected with pCMV6-AC-GFP, pCMV6-AC-GFP-P62, pGFP-V-RS, or pGFP-V-RS-P62. After washing, the bound GTPase is recovered by eluting the GST-fusion protein from the glutathione resin. The purified GTPase is detected by western blot using anti-GTP Ras antibody. The active GTPase population is recovered from the glutathione resin using SDS-PAGE loading buffer and analyzed by western blotting.

### ChIP-3C/ChIP-Loop Assays

The chromatin is cross-linked following the binding to the antibody-protein-A/G-Sepharose beads. The DNA was digested with restriction enzymes and ligated under conditions that favor intramolecular ligation. Immediately after ligation, the chromatin is immunoprecipitated using an antibody (anti-CTCF and anti-RNA polII) against the protein of interest. Samples were then de-cross-linked at 65°C overnight followed by phenol-chloroform extraction and ethanol precipitation. After purification, the ChIP-3C material was detected via PCR with specific primers.

### Cells Proliferation CCK8 Assay

Cells’ proliferation was measured using CCK8 assay kit according to the manufacturer’s instructions (Boshide, Wuhan, China).

### Soft-Agar Colony Formation Assay

Cells were plated on dishes containing 0.5% (lower) and 0.35% (upper) double-layer soft agar. Then, dishes were incubated at 37°C in humidified incubator for two weeks. Soft-agar colonies were stained with 0.05% Crystal Violet for more than 1 hr and counted.

RETRACTED

### Xenograft Transplantation *In Vivo*

The athymic Balb/C mice were purchased from Shi Laike Company (Shanghai, China) and maintained in the Tongji animal facilities approved by the China Association for Accreditation of Laboratory Animal Care. The athymic Balb/C mice were injected in the armpit area subcutaneously with HBMMSCs suspension of 1 × 10^8^ cells in 100 μL of PBS. The mice were observed over 8 weeks and then sacrificed to recover the tumors.

### Histological Analysis

A portion of each tumor was fixed in 4% paraformaldehyde and embedded in paraffin for histological H&E staining according to the manufacturer’s instructions (Qirui, Shanghai, China).

### Statistical Analysis

The significant differences between mean values were obtained from at least three independent experiments. Each value was presented as mean ± SEM. Student’s t test was used for comparisons, with p < 0.05 or p < 0.01 considered significant.

#### Ethics Approval and Consent to Participate

This project was approved by the Ethics Committee of Tongji University. Informed consent was obtained from each patient enrolled in the study. All animal experimental procedures were approved by the Ethics Committee of Tongji University. All methods were carried out in “accordance” with the approved guidelines.

## Author Contributions

Study & Experimental Design, D.D.L.; Experimental Operation & Data Analysis, X.R.X., Z.J.L., Y.N.L., Q.Y.M., C.W., X.N.L., Y.X.Y., J.X., Q.D.Z., X.G., T.M.L., H.P., W.J.W., J.L. and S.J.; Manuscript Preparation, D.D.L.; Manuscript Review & Editing, D.D.L..; Funding Acquisition, D.D.L.

## Conflicts of Interest

The authors disclose no conflicts of interest.

## Supplemental Information

Document S1. Figures S1–S7

Document S2. Article plus Supplemental Information
